The article "Exosomes Derived from Human Bone Marrow Mesenchymal Stem Cells Stimulated by Deferoxamine Accelerate Cutaneous Wound Healing by Promoting Angiogenesis" was retracted in 2023. Reasons: signs of a paper mill; suspected computer-generated content; unreliable results or conclusions; concerns about the data.

# Exosomes Derived from Human Bone Marrow Mesenchymal Stem Cells Stimulated by Deferoxamine Accelerate Cutaneous Wound Healing by Promoting Angiogenesis

**DOI:** 10.1155/2019/9742765

**Published:** 2019-05-05

**Authors:** Jianing Ding, Xin Wang, Bi Chen, Jieyuan Zhang, Jianguang Xu

**Affiliations:** Department of Orthopedic Surgery, Shanghai Jiao Tong University Affiliated Sixth People's Hospital, 600 Yishan Road, Shanghai 200233, China

## Abstract

The exosomes are derived from mesenchymal stem cells (MSCs) and may be potentially used as an alternative for cell therapy, for treating diabetic wounds, and aid in angiogenesis. This study, aimed to investigate whether exosomes originated from bone marrow-derived MSCs (BMSCs) preconditioned by deferoxamine (DFO-Exos) exhibited superior proangiogenic property in wound repair and to explore the underlying mechanisms involved. Human umbilical vein endothelial cells (HUVECs) were used for assays involving cell proliferation, scratch wound healing, and tube formation. To test the effects in vivo, streptozotocin-induced diabetic rats were established. Two weeks after the procedure, histological analysis was used to measure wound-healing effects, and the neovascularization was evaluated as well. Our findings demonstrated that DFO-Exos activate the PI3K/AKT signaling pathway via miR-126 mediated PTEN downregulation to stimulate angiogenesis in vitro. This contributed to enhanced wound healing and angiogenesis in streptozotocin-induced diabetic rats in vivo. Our results suggest that, in cell-free therapies, exosomes derived from DFO preconditioned stem cells manifest increased proangiogenic ability.

## 1. Introduction

Diabetes mellitus has not only seen an increased incidence but the complications associated with this condition have also increased in severity [1]. A ubiquitous and incapacitating impediment in diabetes is decreased diabetic wound healing. This is a medical stumbling block of today that is relevant to patients who either have feet ulcers or are recuperating from complex surgeries that have a possibility of impeding regular activity, chronic ischemic skin lesions, and possible limb amputation of limbs [2]. Wound healing thus depends on an important process of angiogenesis that is involved in delivering nutrition and oxygen to sites of wounds allowing for the proliferation of fibroblasts, synthesis of collagen, and reepithelialization [3]. Healing of wounds, however, gets extended in diabetic patients due to weakened angiogenesis [4]. Diverse biological agents, such as different platelet concentrates, have determined their potential to improve the angiogenesis both in vivo and in vitro [5]. Platelet gel, a recently developed platelet concentrates for topical use, is widely used in different areas of regenerative medicine, such as bone osteoradionecrosis, severe oral mucositis, and wound healing [6, 7]. In order to hasten the process of healing diabetic wounds, the use of new approaches that supplement the local angiogenesis looks promising.

In order to hasten the process of healing diabetic wounds, the use of new approaches that supplement the local angiogenesis looks promising. Mesenchymal stem cells that are multipotent have several potentials for differentiation and immunomodulation [8]. Cell-based therapy appears to be an optimistic therapy for alleviating a worsened diabetic wound. But this direct therapeutic approach still holds risk factors such as the development of tumors and immune responses that are not anticipated [9, 10]. Thus, there is an urgent need to devise new approaches of using stem/progenitor cells that will not have any likely harmful effects because of their direct use and will most effectively realize their therapeutic potential. Several studies have pointed out at a key class of paracrine mediators that function between MSC and target cells: exosomes, which are small particles that are membrane-associated and have an endosomal origin with sizes in the range of 30-150 nm. These mediators bring miRNAs, mRNAs, and proteins to recipient cells and thus have an important part in intercellular communication [11]. Exosomes can be used effectively for direct treatment because they have regenerative attributes like stem cells and may surpass several unwanted effects associated with treatments involving stem cell transplantation. When administered as injections locally, exosomes cause angiogenesis and can promote proliferation and migration of skin cells and closure of wound in animal models with diabetic or burn wound [12, 13], suggesting the exosomes, as a promising therapeutic approach for wound healing.

Stem cells live in niches, which are complex microenvironments, play important roles in directing the function, division, and differentiation of stem cells [14]. Nevertheless, the important approach for in vitro and in vivo enhancement of MSC functions includes preconditioning of MSC culture conditions. The conditions that have shown improvement through tissue engineering and regenerative medicine include cytokines, hypoxia, trophic factors, physical factors, and chemical and pharmacological agents. The hypoxic preconditioning could not only increase the angiogenesis and neuroprotection but also improve proliferation and migration of MSCs, improving the efficiency of the transplantation of MSCs compared to that observed in MSCs under normal culture [15]. Various studies have determined that exosomes derived from mesenchymal stem cells preconditioned by hypoxia own better properties compared with the common MSC-exosome [16, 17]. Preconditioning with other chemical and biological factors could mimic the effect of the hypoxia, such as valproic acid (VPA), CoCl2, deferoxamine (DFO), and dimethyloxaloyl glycine. Various studies have proved that compared with the hypoxia, hypoxia mimetic agent could also induce related hypoxic genes, improving the stemness of MSCs for angiogenesis in studies and clinical tests in a more practically [18–20]. However, hypoxia mimic preconditioned MSCs have not still been used in any research to collect exosomes for being used in therapy. Several hypoxia-response genes have been shown to be induced by an agent, Deferoxamine, that is classical hypoxic-mimetic and mimics the oxygen deprivation effects [21–23].

In this study, we endeavored to study whether exosomes released from BMSCs stimulated by DFO could improve the angiogenic activity in vivo and in vitro and enhance the healing of the impaired diabetic wound.

## 2. Materials and Methods

### 2.1. Cell Culture

Human bone marrow mesenchymal stem cells (BMSCs; ScienCell) were cultured in MEM (Minimum Essential Medium) Alpha Medium (Corning) and 10% fetal bovine serum (FBS, Gibco, NY, USA). BMSCs between passages 4 and 8 were used for the subsequent experiments. Human umbilical vein endothelial cells (HUVECs; ScienCell) were cultured in Endothelial Cell Medium (ECM; ScienCell) containing 5% FBS (ScienCell) and 1% endothelial cell growth supplement (ScienCell). For DFO stimulation, DFO was dissolved in distilled water, which was then diluted in culture medium before use. BMSCs at 80% confluency were incubated for 48 hours in complete medium with exosomes-free FBS and supplemented with 50 *μ*M DFO (Sigma-Aldrich), 100 *μ*M DFO, 200 *μ*M DFO, 400 *μ*M DFO or distilled water as a negative control.

### 2.2. Cell Viability Assay

Cell viability was determined using the cell counting kit-8 (CCK8) assay. The BMSCs were plated at 5000 cells/well into 96-well plates and treated with medium containing 0, 50, 100, 200, and 400 *μ*M of DFO. After 48 hours of incubation, 10 *μ*L CCK8 reagent (Dojindo, Japan) was added to the culture medium and the absorbance of each well was observed at 450 nm by a microplate reader (Bio-Rad 680, Hercules, USA).

### 2.3. Exosomes Isolation

After the harvest of BMSCs conditioned medium, the cells were removed by centrifuging for 10 min at 500 g. Next, the vesicles of apoptosis along with debris were removed by centrifugation of the supernatant for 20 min at 12,000 g and filtering using a filter 0.22 *μ*m pore size. This was followed by ultracentrifugation for 70 min at 110,000 g (Beckman Optima™ XPN, 45Ti) to collect the exosomes in the form of a pellet, which was further resuspended in phosphate-buffered saline (PBS) for further purification by ultracentrifugation for 70 min at 110,000g to remove the contaminating protein. Finally, exosomes were stored at -80°C after being resuspended in PBS. The protein content of exosomes was determined by the Pierce BCA Protein Assay Kit (Thermo Fisher Scientific, USA).

### 2.4. Exosomes Characterization and Internalization

qNano platform (iZON® Science, UK) was used to analyze the distribution and absolute size of the exosomes. The morphological examination of isolated exosomes was done through transmission electron microscopy (TEM; HT7700, Hitachi, Japan). The expression of CD9, CD63, TSG101, and GM130 (the cis-Golgi matrix protein, a negative exosomal marker) in exosomes was evaluated by western blot analysis, and the following primary antibodies were used: CD9, CD 63, TSG101 (1:1000; rabbit IgG, Proteintech and GM130 (1:500; rabbit IgG, Abcam). A green fluorescent dye (DIO; Life Technologies) was utilized to label the exosomes in accordance with the instructions of the manufacturer. Ultracentrifugation at 110,000 g at 4°C for 70 min was performed to remove excess dye. HUVECs were incubated with DIO-labeled exosomes at 50 *μ*g/mL concentration for 8 hours, followed by using of 4,6-diamidino-2-phenylindole (DAPI; Southern Biotech, Birmingham, AL, USA) to stain nuclei and then analyzed by a fluorescent microscope.

### 2.5. Transfection of miRNA Inhibitor

MiR-126 inhibitor and a negative control inhibitor (RiboBio, Guangzhou, China)) at 100 nmol/L were used to transfect BMSCs at 80% confluence with Lipofectamine 2000 in Opti-MEM (Invitrogen) in accordance with the instructions of the manufacturer. After transfection for 5 hours, the cells were cultured in complete medium with or without DFO for 24 h. The supernatant of the culture was used to isolate exosomes.

### 2.6. Real-Time PCR

TRIzol reagent was used for isolation of total RNA from cells while exosomal miRNAs were isolated by using Exosome RNA Purification Kit (Qiagen). For miRNA analysis, the reverse transcription reactions of miRNAs were performed using 4 × Reverse Transcription Master Mix kit (EZBioscience). The qRT-PCR analyses of miRNAs were carried out with FastStart Universal SYBR Green Master (Roche). U6 small nuclear RNA was used to normalize the results.

### 2.7. Western Blot Analysis

Cells were harvested using RIPA lysis buffer, quantified by using the BCA protein assay kit. Protein extracts were separated by sodium dodecyl sulfate-polyacrylamide gel electrophoresis (SDS-PAGE) then transferred to polyvinylidene fluoride (PVDF) membranes. Blocking of membranes was done using 5% nonfat milk for 60 minutes and incubated at 4°C overnight with antibodies against the following proteins: PTEN, p-AKT, AKT (all 1:1000; Abcam), and actin (1:10,000; Thermo Fisher Scientific). Membranes were then incubated with HRP-conjugated anti-rabbit (1:1000) or anti-mouse (1:4000) secondary antibodies (Cell Signaling Technology).

### 2.8. The Assay for Cell Proliferation

Into 96-well plates, HUVECs at 2 × 10^3^ cells/well were seeded. This was followed by the addition of the Exos or DFO-Exos at 50 *μ*g/mL concentration or an equal volume of PBS to the culture medium for 48 h. The proliferation of cells was determined using CCK8 kit. A microplate reader was used to determine the optical density (OD) at 450 nm.

### 2.9. Scratch Wound-Healing Assay

In 6-well plates, HUVECs at 2×10^5^ cells/well were seeded. On reaching confluence, sterile tip of a micropipette was used to make scratch wounds across each well. Each well was washed two times with PBS, and basal medium was added containing Exos or DFO-Exos at 50 *μ*g/mL final concentration. Images for 3 fields of view per scratch were taken at 0h, 24h. The residual fractional wound area was determined and the migratory effect was evaluated using* ImageJ* software.

### 2.10. Transwell Assay

The upper chamber of a 24-well transwell plate (Corning, Corning, NY) was seeded with 5×10^4^ cells. 600 *μ*L of medium supplemented with 50 *μ*g/mL Exos, DFO-Exos, or an equal volume of PBS was added to the lower chamber. After 12 hours of incubation, 0.5% crystal violet was used to stain cells for 5 minutes. A cotton swab was used to remove the cells from the up surface of the membranes after washing thrice with PBS. The number of migrated cells was quantified under an optical microscope (Leica).

### 2.11. Tube Formation Assay

Matrigel from BD Biosciences was used for tube formation assay. In matrigel-coated 24-well plate, 2×10^4^ HUVECs per well were seeded and cultured with 50 *μ*g/mL Exos, DFO-Exos, or an equal volume of PBS for 16 h at 37°C. After 16 h incubation, tube formation was determined under optical microscope (Leica). The total length of the network structures was measured using* ImageJ* software.

### 2.12. Animal Model to Study Skin Wound Healing on Diabetic Rats

250-300 g male Sprague Dawley (SD) rats were used in our study. The Animal Research Committee of the Sixth People's Hospital at the Shanghai Jiao Tong University approved all the procedures. 60 mg/kg of STZ (Sigma-Aldrich, USA) given as one dose intraperitoneally was used to induce diabetes mellitus. Rats with more than 300 mg/dL blood glucose level were chosen for the next stage of the study. Prior to creating wounds in the skin, the diabetic rats were observed for a total of two weeks.

Pentobarbital of 50 mg/kg concentration was injected intraperitoneally to anesthetize STZ-induced diabetic rats. Two excisional wounds of diameter 20 mm were made on the upper back of the rats after shaving, and then they were assigned randomly to three treatment groups. Rats among these groups were administered subcutaneously around the wounds at four injection sites either with Exos (100 *μ*g Exos in 100 *μ*L PBS), DFO-Exos (100 *μ*g DFO-Exos in 100 *μ*L PBS), or 100 *μ*L PBS. The decrease in wound-size was determined: wound-size reduction (%) = (A0 – At)/A0 × 100, where A0 is the area of the wound initially, and At is the area of the wound at week 1 or 2 following wounding.

### 2.13. Microfil Perfusion and Microcomputed Tomography (Micro-CT)

On the 14th day after wounding, rats in three groups were perfused with Microfil (Microfil MV-122, Flow Tech, USA) after anesthetization. For a proper polymerization of the contrast agent, rats were kept at 4°C overnight. The new blood vessels in the wound sites were detected using micro-CT (Skyscan 1176; Kontich, Belgium) for scanning at 9 *μ*m resolution. The original datasets were analyzed by CTAN (Skyscan, Bruker). The threshold is used to distinguish blood vessels from soft tissue by binarization, and the number of blood vessels was quantified.

### 2.14. Histological Analysis

On day 14 after wounding, the skin specimens were fixed in 10 % formalin, dehydrated with a series of graded-alcohol, and embedded in paraffin. After being cut into 4-*μ*m-thick sections, Hematoxylin and eosin (H&E) and Masson's trichrome staining were performed to evaluate extent of wound healing.

### 2.15. Immunohistochemical and Immunofluorescent Analyses

For immunohistochemical analysis, the sections were rehydrated, blocked, and incubated with primary anti-CD31 antibody at 4°C overnight. After incubation with secondary at room temperature, the stained sections were visualized using the DAB substrate and finally counter-stained using hematoxylin.

The formation of blood vessels in granulation tissues was determined at day 14 after wounding by immunofluorescent staining against CD31 and alpha-smooth muscle actin (*α*-SMA). After incubation with Alexa Fluor 488- and Alexa Fluor 594-conjugated secondary antibodies, DAPI was used to stain the nuclei.

### 2.16. Statistical Analysis

Means ± SEM was used to express data. Student's t-test was used for comparing single comparisons. For multiple comparisons, one-way analysis of variance (ANOVA) was performed. A value of P < 0.05 was used as a benchmark for statistical significance.

## 3. Results

### 3.1. Isolation and Characterization of Exosomes

To analyze the optimal working concentration of DFO without impact cell viability in our study, BMSCs were incubated with DFO at concentrations of 0, 50, 100, 200, and 400 *μ*M of DFO. After 48 hours of incubation, the viability of cells was examined by CCK8 assay. The result showed that DFO-treated BMSCs at 100 and 200 *μ*M concentration showed significantly more viability when compared to control group (Figure 1(a)). So, 48 hours treatment with 200 *μ*M of DFO was used to collect DFO-Exos for all experiments in this study.

As presumed, the presence of exosomal marker proteins CD9, CD63, and TSG101 was detected in both Exos and DFO-Exos (Figure 1(b)). qNano analysis was performed to identify Exos and DFO-Exo, finding that the size distribution of most exosomes in two groups was in the range of 50-150 nm (Figure 1(c)). Using TEM analysis, these vesicles with characteristic cup-shaped morphology were observed (Figure 1(d)).

### 3.2. Exosomes Promoted Angiogenesis In Vitro

To determine the activities of exosomes released from BMSCs and DFO-treated BMSCs, we performed an endothelial cell proliferation assay. Compared to the control group, Exos and DFO-Exos enhanced the proliferation of endothelial cell significantly at 24 and 48 hours (Figure 2(a)). And, DFO-Exos exhibited stronger proproliferative effect when compared with Exos group (Figure 2(a)). Transwell assay (Figure 2(b)) and scratch wound-healing assay (Supplementary Figure 1) were used to evaluate the promigratory effects, showing that Exos and DFO-Exos remarkably upregulated the motility of HUVECs while DFO-Exos possessed much stronger promigratory effect that Exos did. Tube formation assay was performed to find that a greater number of cord-like structures were formed on Matrigel in DFO-Exos group, in comparison to the Exos group and control (Figure 2(c)). These results revealed that BMSCs treated with DFO enhance the proangiogenic capacity of exosomes.

### 3.3. Accelerated Wound Healing in Diabetic Rats after Exosomes Treatment

To determine the effects of Exos and DFO-Exos on diabetic wound healing, diabetic rats were established by injection of STZ and full-thickness cutaneous wounds were created on dorsal skin regions, followed by subcutaneous administration of Exos, DFO-Exos or an equal volume of PBS. On days 7 and 14 after wounding, wound closure was accelerated in animals that received Exos treatment in comparison to control PBS, and a higher rate of wound closure was observed in rats treated with DFO-Exos compared with that treated with Exos (Figures 3(a) and 3(b)). H&E staining was carried out to evaluate the extent of wound healing, finding that much longer newly formed epidermis and dermis were observed in the wounds treated with Exos, as compared with wounds in the control group at day 14 after operation (Figure 3(c)). Quantitative analysis confirmed that Exos-treated wounds had a lower level of scar formation than the Exos group (Figure 3(d)). In addition, the further significantly promoted effect on wound healing was observed in DFO-Exos group (Figures 3(c) and 3(d)). Masson's trichrome staining showed the largest amounts of wavy collagen fibers in DFO-Exos-treated-wounds compared to other two groups (Figure 3(e)).

### 3.4. Promoted Angiogenesis in the Wound Sites after Exosomes Treatment

On the 14th day after operation, Microfil perfusion was done to evaluate the blood vessels in the wound sites. The reconstructed 3D images after micro-CT scanning showed a significant increased density of blood vessels after administration of Exos and DFO-Exos, when compared to that in the control group. Additionally, the DFO-Exos-treated wound sites exhibited a greater degree of formation of blood vessels (Figure 4(a)). Immunohistochemical staining against CD31 and immunofluorescence double-staining for CD31 and *α*-SMA were done to identify the blood vessels in wound sites that received various treatment. According to the results, the number of overall (Figure 4(b)) as well as mature blood vessels (Figure 4(c)) in the wound sites that received DFO-Exos and Exos treatment was enhanced remarkably compared to that in the control group, and a larger number of these two parameters were identified in the DFO-Exos group, when compared to that in Exos group (Figures 4(c) and 4(d)). These results revealed that DFO pretreatment enhances BMSCs-derived exosomes mediated angiogenesis in wound healing.

### 3.5. Exosomal Transferred-miR-126 from BMSCs Is Promoted to Activate PI3K/AKT Pathway after DFO Treatment

Quantitative real-time PCR (qRT-PCR) was utilized to examine the levels of key proangiogenic miRNAs, such as miR-214, miR-21, miR-126, miR-125b, miR-27b, and miR-19b in exosomes. Among these detected miRNAs, miR-126 was found to display marked upregulation after DFO treatment (Figure 5(a)). Next, we determined whether Exos or DFO-Exos could be internalized into HUVECs, cause internalization is an essential condition for transfer of miRNAs via exosomes. Exos and DFO-Exos were labeled by the green fluorescent dye (DIO) and then were incubated with HUVECs for 8 hours. Fluorescence microscopy confirmed that DIO-labeled Exos and DIO-labeled DFO-Exos had been transferred to perinuclear region of HUVECs (Figure 5(b)). To verify the transfer of miR-126, HUVECs were treated with Exos and DFO-Exos. Then the cells from different groups were harvested for PCR analysis. As shown in Figure 5(c), miR-126 levels in HUVECs were significantly increased after the cells were incubated with Exos and DFO-Exos for 3 hours respectively, and the level of miR-126 was higher significantly in DFO-Exos-treated HUVECs. Studies have shown that miR-126 can target PTEN in cells to induce the activation of PI3K/AKT pathway. Analysis by western blot in HUVECs after different treatments showed much more reduction of phosphatase and tensin homolog (PTEN) and an increase in the amount of phosphorylation of AKT (p-AKT) in cells subjected to DFO-Exos treatment, when compared to that in Exos and control groups (Figure 5(d)). These results suggested that exosomes released from BMSCs by DFO stimulation directly by more miR-126 to endothelial cell by activating PI3K/AKT pathway.

Then, BMSCs were transfected with miR-126 inhibitor or negative control inhibitor before DFO stimulation, as shown in Figure 6(a), and the miR-126 level was significantly inhibited in DFO-treated BMSCs-derived exosomes (126I-DFO-Exos). To explore the effects of exosomes derived from miR-126 knockdown DFO-BMSCs, western blot analysis showed that PTEN was upregulated and p-AKT was downregulated in 126I-DFO-Exos group (Figure 6(b)). The transwell assay showed that the number of migrated cells in the group treated with miR-126 knockdown DFO-Exos was significantly decreased (Figure 6(c)), as well as the length of tubes and branch numbers in the 126I-DFO-Exos group determined by tube formation assay (Figure 6(d)). These results suggested that miR-126 plays the vital role in the enhanced proangiogenic effect of exosomes from DFO-stimulated BMSCs.

## 4. Discussion

In this study, we investigated exosomes derived from MSCs preconditioned by DFO which exhibit superior proangiogenic properties in vitro and in vivo. The results in this study show that, in presence of DFO-Exos, the levels of miR-126, a proangiogenic component, were enhanced remarkably in the HUVECs. Furthermore, in the diabetic skin wound animal model, the proangiogenic effects of exosomes were increasingly mediated by miR-126.

Preconditioning using hypoxia causes an increase in angiogenesis induced by MSCs as well as alterations of mRNA and proteins in exosomes; furthermore, interactions between these exosomes and endothelial cells boosted the angiogenic potential of the latter, according to several studies [16, 24, 25]. This current work involved an isolation of exosomes from BMSCs that were exposed to a pretreatment of DFO that displayed greater proangiogenic properties in vitro. A direct communication between the exosomes and their target cells in order to deliver particular miRNAs and proteins prototypical of the origin of the exosomes is thought to be the mechanism of angiogenesis mediated by exosomes [17]. The levels of miR-296, miR-21, and miR-126 that are vital microRNAs involved in angiogenesis were evaluated in our study. A surprising observation was an elevation of significance in levels of miR-126 in DFO-Exos. The levels of this miRNA were increased in the HUVECs after the treatment by the DFO-Exos. A vital role has been implicated for miR-126 in development of vascular tissues [26]. Concurrently, exosomes released by CD34b peripheral blood mononuclear cells also contain miR-126, which regulates angiogenesis after being transferred to endothelial cells [27]. This is the first study that reports an upregulation of expression of miR-126 in exosomes derived from MSCs by stimulation by DFO and exhibits higher effects of proangiogenesis in vitro and in vivo.

In addition, it was also observed that the quantity of an established target of the miRNA: PTEN was lowered in endothelial cells when DFO-Exos were administered while the levels rose when miR-126 was inhibited. This is suggestive of a regulation of expression of the target in endothelial cells by microRNA uptake. The proangiogenic pathway is inhibited in endothelial cells by PTEN through PI3K/AKT signaling to suppress growth factor signaling [26]. Along the same lines, the HUVECs cultured with DFO-Exos showed elevated levels of phosphorylation of AKT while the level was lower in HUVECs that were cultured with exosomes that had inhibited miR-126. These results are indicative of proangiogenic functions of exosomes from MSCs that are released by DFO stimulation.

In conclusion, our study showed that MSC derived exosomes stimulated by DFO in low doses promote neovascularization via the PI3K/AKT pathway and enhance skin wound recovery in the diabetic skin wound animal model. Thus, DFO may cause exosomes to be triggered in order to show augmented proangiogenic potential in cell-free therapeutic applications.

## Figures and Tables

**Figure 1:** Characterization of exosomes. (a) Viability assay of BMSCs treated with various concentrations of DFO for 48 hours. DFO-treated BMSCs at 100 and 200 *μ*M concentration showed significantly more viability when compared to control group. ^*∗∗∗*^ P < 0.001 versus control. (b) Western blotting showed the presence of exosomal markers including CD9, CD63, and TSG101 in Exos and DFO-Exos. (c) qNano analysis results of Exos and DFO-Exos. (d) TEM photomicrographs of Exos and DFO-Exos. Scale bar = 50 nm.

**Figure 2:** The proliferation and proangiogenic effects of Exos and DFO-Exos on HUVECs. (a) Proliferation of HUVECs treated with Exos or DFO-Exos at 50 *μ*g/mL concentration or an equal volume of PBS. ^*∗∗∗*^ P < 0.001 versus control, ^###^ P < 0.001 versus Exos group. (b) Left panel, representative images of transwell assay, scale bar = 200 *μ*m; right panel, quantitative analysis of the assay. ^*∗∗∗*^ P < 0.001 versus control, ^###^ P < 0.001 versus Exos group. (c) Left panel, representative images of tube formation assay from three groups, scale bar = 200 *μ*m; right panel, quantitative analysis of the assay. ^*∗∗∗*^ P < 0.001 versus control, ^###^ P < 0.001 versus Exos group.

**Figure 3:** Cutaneous wound healing in diabetic rats is accelerated after Exos and DFO-Exos transplantation. (a) Gross view of wounds treated with Exos, DFO-Exos or PBS on days 0, 7, and 14 after wounding. (b) The wound-closure rates on specific days of three groups. ^*∗∗∗*^ P < 0.001; ^*∗∗*^ P < 0.01 versus control, ^###^ P < 0.001 versus Exos group. (c) H&E staining of wound sections from three groups at 14 days after wounding. The black arrows point out the scar edges. Scale bar = 1000 *μ*m. (d) Quantitative analysis of the scar widths. ^*∗∗∗*^ P < 0.001 versus control, ^###^ P < 0.001 versus Exos group. (e) Masson's trichrome staining for the evaluation of collagen maturity. Scale bar = 100 *μ*m (top) or 50 *μ*m (bottom).

**Figure 4:** Promoted angiogenesis in the wound sites after exosomes treatment. (a) Left panel, Microfil perfusion for determination of blood vessel density in the wound sites on day 14 after wounding; right panel, quantitative analysis of blood vessel density in three groups. ^*∗∗∗*^ P < 0.001 versus control, ^###^ P < 0.001 versus Exos group. (b) Left panel, immunohistochemical staining against CD31 of wound sections on day 14 after wounding. Scale bar = 50 *μ*m; right panel, quantitative determination of the number of total blood vessels. ^*∗∗∗*^ P < 0.001 versus control, ^###^ P < 0.001 versus Exos group. (c) Left panel, immunofluorescent staining against CD31 and *α*-SMA of wound sections from three groups on day 14 after wounding. Scale bar = 50 *μ*m; right panel, quantitative determination of the number of mature blood vessels. ^*∗∗∗*^ P < 0.001 versus control, ^###^ P < 0.001 versus Exos group.

**Figure 5:** DFO-Exos deliver more miR-126 into the endothelial cells. (a) The levels of angiogenic miRNAs among Exos and DFO-Exos were determined by qRT-PCR. ^*∗∗*^ P < 0.01 versus Exos group. (b) Fluorescent microscopy showed the internalization of DIO-labeled Exos of DFO-Exos by HUVECS. Exosomes could be seen in the perinuclear region of HUVECs. Scale bar = 20 *μ*m. (c) The level of miR-126 in HUVECs after DFO-Exos, Exos, or PBS treatment was evaluated. ^*∗∗∗*^ P < 0.001 versus control, ^###^ P < 0.001 versus Exos group. (d) Western blotting analysis of PTEN, p-AKT, and AKT expression in HUVECs among three groups.

**Figure 6:** Effects of DFO-Exos with miR-126 knockdown on angiogenesis of endothelial cells. Levels of miR-126 in exosomes from BMSCs treated with DFO + PBS (DFO-Exos), DFO + negative inhibitor control (NCI-DFO-Exos), or DFO + miR-126 inhibitor (126I-DFO-Exos) were analyzed by qRT-PCR. ^*∗∗∗*^ P < 0.001 versus DFO-Exos, ^###^ P < 0.001 versus NCI-DFO-Exos group. (b) Western blotting analysis of PTEN, p-AKT, and AKT expression in HUVECs among three groups. (c) Left panel, representative images of transwell assay, scale bar = 200 *μ*m; right panel, quantitative analysis of the assay. ^*∗∗∗*^ P < 0.001 versus DFO-Exos, ^###^ P < 0.001 versus NCI-DFO-Exos group. (d) Left panel, representative images of tube formation assay from three groups, scale bar = 200 *μ*m; right panel, quantitative analysis of the assay. ^*∗∗∗*^ P < 0.001 versus DFO-Exos, ^###^ P < 0.001 versus NCI-DFO-Exos group. (e) Schematic diagram depicts the enhanced proangiogenic effects of DFO-Exos on wound healing. Followed by subcutaneous administration of DFO-Exos, Exos, or PBS, higher rate of wound closure was observed in rats treated with DFO-Exos due to the improvement of angiogenesis.

## Data Availability

The data used to support the findings of this study are available from the corresponding author upon request.

## Supplementary Materials

Supplementary Materials Supplementary Figure 1. The promigratory effects of Exos and DFO-Exos on HUVECs. Left panel, scratch wound-healing assay of HUVECs treated with Exos or DFO-Exos at 50 *μ*g/mL concentration or an equal volume of PBS, scale bar = 200 *μ*m; right panel, quantitative analysis of the assay. ^*∗∗∗*^ P < 0.001 versus control, ### P < 0.001 versus Exos group.
